The article "Application of Apriori Improvement Algorithm in Asthma Case Data Mining" was retracted in 2023. Reasons: signs of a paper mill; compromised peer review; unreliable results or conclusions.

# Application of Apriori Improvement Algorithm in Asthma Case Data Mining

**DOI:** 10.1155/2021/9018408

**Published:** 2021-11-01

**Authors:** Yi Zheng, Peipei Chen, Biyu Chen, Dengjun Wei, Meifang Wang

**Affiliations:** Department of Respiratory and Critical Care Medicine, Taihe Hospital, Hubei University of Medicine, Shiyan 442000, Hubei Province, China

## Abstract

In Chinese medicine, asthma cases contain a large amount of empirical data which are obtained from the clinical diagnosis of doctors throughout the year. Data correlation analysis method is among the common mechanisms which are used to mine association between the (1) prescriptions and prescribers (doctors in this case) and (2) symptoms and medications for a particular disease in the hospitals. In this paper, initially, a thorough analysis of expected performance and shortcomings of the Apriori algorithm in mining of medical case data is presented. Secondly, we propose an extended version of the traditional Apriori algorithm which is primarily based on the fast response of computer to bit-string logic operation. A comparative evaluation of the proposed and existing Apriori algorithms is presented particularly in terms of running time, mining of frequent items set and strong association rules. Both experimental and simulation results have proved that the proposed extended Apriori algorithm has outperformed existing algorithms when it is applied to asthma medication and combined symptom-medication data for the association analysis. Furthermore, the association relationship between mind asthma case data and medication is effective in the analysis of asthma case data with significant application value which is verified by the experimental data and observations.

## 1. Introduction

Due to the rapid development in the Internet of Medical Things (IoMT), particularly wearable devices such as sensor and actuator, the smart healthcare systems continue to expand and generate a large amount of data every day. To cope with this huge data values, association rule is among the common approaches in the literature. Association rule mining refers to the mining of interest between different elements of a particular data set, and these rules are generally valuable for the exploitation. The Apriori algorithm provides new ideas to extend existing association rule mining to an acceptable and generalized version. For example, Ye [1] has designed an algorithm based on negation rules to enhance accuracy and precision of the proposed system. Likewise, Zhou and Tian [2] have proposed an algorithm based on interest degree association rules whereas Shao [3] has proposed a frequent item set mining algorithm based on matrix and item set index table. Wang et al. [4] have successfully used an optimized association rule that is the Apriori algorithm. Sleep apnea hypoventilation syndrome is a common clinical respiratory disease, and intelligence-assisted medical modeling is a potential platform for mining medical data to achieve medical assistance [5, 6]. Modern data analysis techniques are used to analyze the patient's basic information, medical history, physical condition, and other important textual characteristics of potential causes. Furthermore, relationship with PSG examination results, role of potential causes on the onset, severity, progression, and prognosis of obstructive sleep apnea patients, and their interaction mechanisms are thoroughly examined to achieve automatic medical clinical assistance and become the current diagnosis of the condition [7].

The article "Application of Apriori Improvement Algorithm in Asthma Case Data Mining" was retracted in 2023. Reasons: signs of a paper mill; compromised peer review; unreliable results or conclusions.

In the literature, a single established model for sleep apnea hypopnea syndrome (PSG) is not available yet, and majority of the diagnosis are performed manually using traditional experience which inevitably leads to misdiagnosis and is a time consuming process as well. In order to solve these problems, the existing Apriori algorithm was studied extensively and a medical model of sleep apnea hypoventilation syndrome based on the improved Apriori algorithm was developed as a potential candidate solution. Validity of this model was verified by using the medical records (cases) of sleep apnea hypoventilation syndrome which was provided by the hospital. In the real world, there are usually interdependent or interrelated relationships between things, and when something is already known, the things that are related or dependent on it can be inferred, and the rules that express such related or dependent relationships between things are called association rules [8]. At present, association rules have important applications in different fields. Throughout this study, multidimensional association rules are used to analyze the impact of different months, regions, sectors, and other factors on debt and earnings. Moreover, it is an important application of association rules in the field of finance. In the retail industry, association analysis is used to examine customer demand, product sales, trends, and fashions along with mining rules to maximize the expected profits. Likewise, in the telecommunications industry, association rules are used to perform analysis of customer demand, product sales, and product trends and fashions and to maximize profits. In the retail industry, correlation analysis is utilized to identify customer needs, product sales, as well as product trends and fashions, mine rules, and then rationalize the mix and placement of products to maximize the profits. Likewise, in the telecommunication industry, correlation analysis is very helpful to grasp business trends, identify which telecommunication model is more effective, and capture some misappropriation. It is carried out to utilize the available resources in a more effective manner and thus improve quality of services. Chinese asthma cases [9] contain a large amount of empirical data which are collected from the clinical diagnosis of physicians. Correlation analysis mechanism is a potential candidate method to represent these data in the form of knowledge, which is important for the objectification of Chinese medicine data and transmission of physicians' experience and medical research [10, 11].

The article "Application of Apriori Improvement Algorithm in Asthma Case Data Mining" was retracted in 2023. Reasons: signs of a paper mill; compromised peer review; unreliable results or conclusions.

In this paper, we have initiated a thorough evaluation of the classical Apriori algorithm particularly through flowchart and examples. Secondly, we have proposed an enhanced version of the traditional Apriori algorithm which is based on bit logical operation, that is, Apriori-BSO algorithm. Furthermore, the proposed algorithm was used in the association analysis of asthma case data and mined successfully the valuable data rules in asthma diagnosis and treatment process. Main contributions of this paper are presented as follows:

1. An enhanced Apriori-based algorithm to ensure effective mining of the asthma diagnosis and treatment data values
2. A bit logical operation-based Apriori-BSO algorithm for the smart healthcare systems particularly for diagnosis and mining purposes
3. Thorough evaluation of the traditional Apriori algorithm and its weaknesses particularly from diagnosis and mining perspective

The remaining paper is organized as follows. In the subsequent section, that is, Section 2, a comprehensive description of the association rules is presented which is followed by proposed system or algorithm working methodology preferably in detailed and more understandable form. In Section 4, a detailed description of the comparative analysis of the proposed and existing algorithm in terms of numerous performance metrics is presented. Finally, concluding remarks and future directives are given at the end of the manuscript.

## 2. Basic Concepts of Association Rules

Association rules are defined as set rules which describe how various entities or things are associated with each other. To understand this phenomenon, let us define A as a set of items, called an item set. If the item set A contains *k* items, then it is called the *k* item set. The number of occurrences of item set A and the total number of transactions in transaction database D are counted and the number of occurrences divided by the total number of transactions is the support of the item set [12]. If the support of the item set is greater than a predefined threshold values, then item set is called a frequent item set.

The article "Application of Apriori Improvement Algorithm in Asthma Case Data Mining" was retracted in 2023. Reasons: signs of a paper mill; compromised peer review; unreliable results or conclusions.

An association rule represents an association between things and can be expressed by an equation like *X* and *Y* where *X* = I and *Y* = I, and *X* ∩ *Y* = I is the set of all items in D. If the percentage of *X* ∪ *Y* in the transaction database D is s%, then the support of the association rule XY is said to be s%, and in fact, the support is the probability value. The support of the set of items *X* is expressed as follows:

(1) $$\begin{array}{c} \text{support }\left(X⟶Y\right)=P\left(XUY\right). \end{array}$$

Likewise, the confidence of the rule is expressed as follows:

(2) $$\begin{array}{c} \text{confidence }\left(X⟶Y\right)=P\left(\frac{X}{Y}\right). \end{array}$$

In fact, confidence is a conditional probability *P*(*Y*/*X*). Furthermore, support and confidence values are calculated by utilizing equations (1) and (2), repectively. That is, a relationship between things is called an association rule if it satisfies a predetermined confidence and support level.

## 3. Traditional Apriori Algorithm

The traditional Apriori algorithm (prior knowledge about items) is used to find ratio of the frequent item set in a given data set. It is to be noted that the Apriori algorithm assumes that every nonempty subset of the concerned frequent set should be frequent. Apart from it, if an item is assumed to infrequent, then it is high likely that its superset must be infrequent as well.

### 3.1. Performance Analysis of the Traditional Apriori Algorithm

As described above, the Apriori algorithm is mainly the process of discovering frequent itemsets in a given data set, and those frequent itemsets contained in the transaction are only accounted for a small portion. To avoid calculating the support of all itemsets and generating a large number of calculations, in the Apriori algorithm, the known frequent itemsets are used to generate itemsets of longer length, called candidate frequent itemsets. Furthermore, the frequent itemsets are obtained by filtering the candidate frequent itemsets [13]. The process of generating frequent itemsets is based on the following property; that is, the subset of frequent itemsets must be frequent itemsets. The steps of Apriori algorithm are as follows [14]:

(1) *Scan the Database D Once*. The support count of each itemset is counted (the support count of an item set is the number of times the item set appears in the database), and the item set that meets the minimum support threshold is added to the frequent item set *L*_1_.
(2) *Join Step.* The JOIN operation, which generates a candidate *k* item set from the items in the frequent (*k*−1) item set *L*_*k*−1_, is the join step, i.e., the JOIN operation that is represented as follows:
  (3) $$\begin{array}{c} O_{p,q}\;\in \;L_{k-1},\\ p=\left\{p_{1},\;p_{2},\;\ldots \ldots p_{k-2},\;p_{k-1}\right\},\\ q=\left\{q_{1},\;q_{2},\;\ldots \ldots q_{k-2},\;q_{k-1}\right\}. \end{array}$$
When 1 ≤ *i* < *k* − 1, *p*_*i*_=*q*, and when *i*=*k* − 1 and *p*_*k*−1_ ≠ *q*_*k*−1_, then
  (4) $$\begin{array}{c} p\cup q=\left\{p_{1},\;p_{2},\;\ldots \ldots p_{k-2},\;p_{k-1}\right\}, \end{array}$$
is added to the set *C*_*k*_ of the candidate frequent *k* item set.
(3) *PuningStep*. The itemsets in *C*_*k*_ are not all frequent, and the candidate frequent itemsets are too large to bring a large computational overhead to the operation of the algorithm. Therefore, it is necessary to delete these itemset which is based on the following principles:
  If (*k*−1) itemset is not frequent, then the *k* itemset containing it must not be a frequent *k* itemset, so when the candidate *k* itemset has a (*k*−1) itemset that is not in *L*_*k*−1_, then the candidate *k* itemset is not frequent and should be removed from *C*_*k*_.
(4) The database D is scanned once, and the support of each item set in *C*_*k*_ is calculated.
(5) By comparing the support thresholds, the candidate *k* itemset *C*_*k*_ is removed from the set of items smaller than the support threshold and the remaining item sets from the set of frequent *k* itemsets *L*_*k*_.

Run Steps 2 to 5 repeatedly until new set of frequent item sets cannot be generated. From the above steps, we have concluded that the traditional Apriori algorithm generates all frequent item sets that satisfy the minimum support threshold values in a given application domain.

The article "Application of Apriori Improvement Algorithm in Asthma Case Data Mining" was retracted in 2023. Reasons: signs of a paper mill; compromised peer review; unreliable results or conclusions.

According to the steps of the Apriori algorithm, the operational flow of the traditional Apriori algorithm is quite similar to that the once presented in Figure 1.

From the operation or execution order of the traditional Apriori algorithm, we have observed that it has various limitations in terms of time consumption, that is, (1) the process of generating frequent itemsets from candidate itemsets is a multitrip scan of the massive database and (2) the joining of *k*−1 frequent itemsets with *k*−1 frequent itemsets when using the JOIN step to generate candidate itemsets needs to ensure that the *k*−2 and *k*−1 items are the same and different, respectively. This process also increases the computational cost of the algorithm, and the candidate itemsets generated by the JOIN step are large and increasing as the number of frequent 1 itemsets increases. For example, if there are five (5) frequent 1 itemsets, then there are 10 candidate 2 itemsets; if there are 1000 frequent 1 itemsets, then the candidate 2 itemsets will be *C*_1000_^2^; and if there are 10000 frequent 1 itemsets, the candidate 2 itemsets will be *C*_10000_^2^, as many as 10^7^, which is a very large amount of computation [10].

### 3.2. Proposed Enhanced Apriori Algorithm

One of the challenging issues associated with the traditional Apriori algorithm is that it has to scan the database multiple times and generate a large set of candidate items. To resolve this issue, an enhance version of the traditional Apriori algorithm, which is based on the bit-string logic algorithm and called the Apriori-BSO algorithm, is presented. The proposed enhanced Apriori algorithm, which is based on the logical operation of bit string, is primarily designed for the fast response of computer to the bit string, using the concept of “bit” in mathematics [15] where each individual thing I in the thing database D is represented by a bit string. According to the logical operation of “fit” to find the support count of the item set [16], combined with the classical Apriori algorithm [17], the frequent item set and strong association rules are mined. Numerous possible steps, specifically mandatory steps, of the whole algorithm are as presented as follows:

1. Support and confidence threshold values are set.
2. The database is scanned, and “1” and “0” are used to indicate whether each item in the transaction library appears in the transaction or not. In scenarios where it appears, it is recorded as “1,” and if it does not appear, then recorded as “0.” The occurrence of each item in the transaction library is represented as a set of bit strings. The number of “1” in the bit string corresponding to each item is counted, which is the support count of the item. Candidate items to support counts are greater than the threshold that is selected as the items in the frequent 1 item set *L*_1_.
3. An item sequence S is generated according to *L*_1_, *S* = the set of item bit strings in *L*_1_. Each item is coded to generate a coded bit string: the length of the code is the number of items in the library, and if a single item appears in the generated set of items, the position of the corresponding item sequence is recorded as “1”; otherwise, it is “0.”
4. The concatenation operation is performed on *L*_*k*−1_. Logical “or” operations are performed on the item code bit strings in *L*_*k*−1_, and the number of “1s” in the resultant bit strings is counted; if it is *k*, it will be added to the candidate *k* item set *C*_*k*_.
5. A logical “and” operation is performed on the item bit string of *L*_*k*−1_ corresponding to the item in the generated *C*_*k*_. The final result is the item bit string of the corresponding item in *C*_*k*_. The number of “1” in the item bit string is the support count of the candidate. The candidate item whose support count is greater than the threshold is regarded as the item in the frequent *K* item set *L*_*k*_. The above steps are repeated, and the algorithm is stopped until the number of single items contained in *L*_*k*_ is less than (*K* + 1).

The article "Application of Apriori Improvement Algorithm in Asthma Case Data Mining" was retracted in 2023. Reasons: signs of a paper mill; compromised peer review; unreliable results or conclusions.

The operation flow of the algorithm is shown in Figure 2.

Properties of the algorithm are as follows:

 
*Property 1.* A subset of a frequent k-term set must also be frequent
 
*Property 2*. If the number of single items in a frequent *k* item set is less than (*k* + 1), the set of frequent (*k* + 1) items is not generated

## 4. Simulation Results and Performance Evaluation of the Proposed Enhanced Apriori Algorithm

To verify the exceptional performance of the proposed enhanced Apriori algorithm, it and existing schemes are implemented in java. These algorithms were tested on large and benchmark data set under the same conditions, i.e., data set size, computational power, and resources. Benchmark data sets are provided by the UCI directory, which is openly available online. The proposed enhanced Apriori-BSO algorithm simulation results were compared with that of the traditional Apriori algorithms as shown in Figure 3. It is evident from the simulation results that the proposed scheme is an ideal solution particularly for the application area where minimum possible running time of machine or devices is preferred. The results demonstrate that the running time of the proposed enhanced apriori-based algorithm has decreased significantly than that of the classical algorithm as the number of processed data records increases in the benchmark or real-time data sets.

From Figures 4 and 5, we have concluded that the proposed enhanced Apriori algorithm, which is based on the combination idea, has performed exceptionally well when the width of a single data set is small in the given benchmark data set. The enhanced Apriori algorithm based on bit-wise operations and preparing performs better than traditional algorithms when the width of a single data set is large and the exceptional performance is likely to continue more and more which is obvious as the width increases. Furthermore, we have concluded from the simulation results that accuracy of apriori-based algorithms is approximately 100%.

In dataset 1, asthma images were acquired from a wide range of sources and in a variety of ways. Some images contain multiple asthma regions and multiple asthma samples, but some images contain only one asthma region and the background region. This has an impact on the classification and recognition of the images. To verify the performance of the proposed model, an image containing multiple asthma regions was set up for classification, and the classification results are shown in Figure 6, with an average accuracy of 97%, indicating that the proposed model has good learning ability and mine successfully the feature differences between asthma diseases. It also illustrates the reliability and practicality of the collected data as well.

The article "Application of Apriori Improvement Algorithm in Asthma Case Data Mining" was retracted in 2023. Reasons: signs of a paper mill; compromised peer review; unreliable results or conclusions.

The accuracy rates of the four networks are shown in Table 1.

As shown in Table 1, compared with the benchmark method, the accuracy of asthma identification in different banks is improved by 6% and the identification is better by the proposed models. Additionally, the performance of the latest models is not as good as the proposed enhanced apriori-based model because existing models do not have the detailed grasp of different regions or asthma. Asthma characters in the asthma images are first projected horizontally to obtain the boundaries; the different views of asthma are input to different channels of our model, and different training methods are still used for different practical applications. Compared with a single ResNet, the proposed method is more efficient. Thus, the proposed model has learned image features from the image element level, which is an advantage of the model on the one hand, and thanks to the proposed feature processing of image boundaries on the other hand.

As shown in Figure 7, the loss ratio of the proposed method decreases rapidly during the training period and the loss is smooth in the subsequent training iterations. The results show that the proposed model is stable and converges quickly. This model is trained from 11 epochs, which is due to the establishment of the multichannel integrated learning method, which enables this model to learn simple knowledge quickly and effectively. As shown in ResNet and annexed, although these algorithms start training from 20 epochs, these models are unstable and the loss shows local oscillations, which is due to the fact that a single model cannot handle images from different angles well and lacks robustness.

### 4.1. Excavation Results

In medical data set, the individual data width is 39; thus, we have decided to experiment with medical case data and analyze the results using the proposed enhanced Apriori algorithm based on bit-wise operations and preparing. The results presented in Table 2 are some of the sets of transactions that lead to sleeping apnea hypoventilation syndrome and their support.

### 4.2. Analysis of Mining Results

In these results which are presented in Table 2, it is clear that the causes of sleep apnea hypoventilation syndrome and its susceptible groups are as follows:

1. Most of the patients are male, basically they have symptoms of snoring at night. Additionally, most of them have symptoms such as dry mouth in the morning and drowsiness during the day, most of them have irregular life and rest, and some of them have family history of the disease.
2. Young men, who snore in bed, are drowsy during the day. They interfere with their work and generally show slight excessive sleepiness as these men are highly susceptible group.
3. Men with easy to wake up at night, drowsiness during the day, dry mouth in the morning, and snoring in bed were the susceptible group.

The article "Application of Apriori Improvement Algorithm in Asthma Case Data Mining" was retracted in 2023. Reasons: signs of a paper mill; compromised peer review; unreliable results or conclusions.

The above results are consistent with clinical performance, indicating that the given model is valid and have provided relevant data for realizing rapid real-time online diagnosis of numerous patients.

## 5. Conclusion and Future Work

In this paper, we have thoroughly analyzed the performance and shortcomings of the classical Apriori algorithm and the proposed enhanced Apriori algorithm based on the fast response of computer to bit-string logic operation. Additionally, we have compared running time of the these algorithms under the same conditions in java. For this purpose, we have normalized the collected asthma medical case data and used the enhanced Apriori algorithm to correlate the asthma medication data and symptom-medication combination data and mined out the rules of asthma medical prescription dispensing pattern and the correlation between symptoms and medication. Association analysis of asthma medication data and combined symptom-medication data was performed by the enhanced Apriori algorithm, and the association between asthma prescriptions and symptoms and medication was mined.

In future, we are planning to improve the performance of the proposed enhanced Apriori algorithm by integrating smart and intelligent deep learning-based models.

## Figures and Tables

**Figure 1:** Flow chart of the Apriori algorithm.

**Figure 2:** Priori BSO algorithm flow chart.

**Figure 3:** Comparison of the running time of the Apriori-BSO algorithm and classical Apriori algorithm.

**Figure 4:** Algorithm running time curve with data length.

**Figure 5:** Algorithm running time curve with data width.

**Figure 6:** Effect of asthma classification.

**Figure 7:** Convergence effect of multiview asthma model training.

**Table 1:** The accuracy of each method.

Type of network	Training set (%)	Test set (%)
CNN	76.23	76.16
AlexNet	80.45	79.58
ResNet	81.56	80.23
Proposed method	83.21	82.40

**Table 2:** Partial mining results.

Number of items	Itemset	Support
5	Male snores, wakes up at night, sleepy during the day, dry mouth in the morning	22.459
5	Male complained of snoring, sleepiness during the day, and dry mouth in the morning	22.836
5	Male complained of snoring, suffocating at night, and dry mouth in the morning	22.961
5	Young men affect work and daytime sleepiness Epworth 3	25.345
5	Male complained of dry mouth in the morning and his parents had a history of snoring	20.075
4	Snore, hold up at night, dry mouth in the morning, and have a history of drinking	20.201
4	Male sleepy during the day, dry mouth in the morning, and a history of drinking	20.326
4	Male dry mouth in the morning and diastolic blood pressure in the morning Epworth 2	20.452
4	The chief complaint was snoring, waking up at night, and sleepiness during the day	20.577
4	Male daytime sleepiness youth daytime sleepiness	20.577
4	Snoring, sleepiness during the day, dry mouth in the morning, and drinking history	20.703
4	Male complained of snoring and dry mouth in the morning	34.253

The article "Application of Apriori Improvement Algorithm in Asthma Case Data Mining" was retracted in 2023. Reasons: signs of a paper mill; compromised peer review; unreliable results or conclusions.

## Data Availability

The datasets used and analyzed during the current study are available from the corresponding author upon reasonable request.
